# Safety of Anlotinib Capsules Combined with PD-1 Inhibitor Camrelizumab in the Third-Line Treatment of Advanced Non-Small-Cell Lung Cancer and Their Effect on Serum Tumor Markers

**DOI:** 10.1155/2021/2338800

**Published:** 2021-12-15

**Authors:** Yinhua Wang, Xiuhua Shi, Qinghua Qi, Bin Ye, Zhaoling Zou

**Affiliations:** ^1^Department of Radiotherapy, The Second People's Hospital of Wuhu City, Wuhu, 241000, Anhui Province, China; ^2^Department of Hematology, The Second People's Hospital of Wuhu City, Wuhu, 241000, Anhui Province, China

## Abstract

**Objective:**

To explore the safety of anlotinib capsules combined with the PD-1 inhibitor (camrelizumab) in the third-line treatment of advanced non-small-cell lung cancer (NSCLC) and their effect on serum tumor markers.

**Methods:**

88 patients with advanced NSCLC treated in the Oncology Department of our hospital from December 2018 to December 2019 were selected as research subjects and randomly and equally split into the single treatment group (STG) and combined treatment group (CTG). The levels of serum tumor markers after treatment were detected in both groups, and the incidence of adverse reactions during treatment was recorded.

**Results:**

Compared with the STG, CTG achieved obviously higher total effective rate (*P* < 0.05), lower total incidence of adverse reactions (*P* < 0.05), lower levels of serum tumor markers and average CFS score (*P* < 0.001), and higher average KPS score (*P* < 0.001).

**Conclusion:**

Application of anlotinib capsules combined with the PD-1 inhibitor (camrelizumab) in the third-line treatment of advanced NSCLC can effectively reduce the levels of serum tumor markers and cancer fatigue degree of patients, with a better effect than that of simple anlotinib treatment. In addition, further research of the combined treatment is helpful to establish a better therapeutic regimen for patients with advanced NSCLC.

## 1. Introduction

With the changes in people's lifestyle and environment, the incidence of lung cancer in China has increased [1]. Radical resection of lung cancer is the best treatment for this disease. However, due to the occult onset of the cancer, most patients have entered the advanced stages when diagnosed, missing the best surgery time. Therefore, they turn to systemic chemotherapy, immunotherapy, or molecular targeted drug therapy [2–4]. Non-small-cell lung cancer (NSCLC) has a high incidence, accounting for about 65–80% of lung cancer, and the chemotherapy drugs are mostly cytotoxic drugs, which can fight against cancer and reduce tumors by damaging the DNA structure and affecting nucleic acid synthesis, but can trigger adverse reactions such as gastrointestinal reactions and myelosuppression because they do not have specificity for tumor cells and have a lethal effect on normal cells [5–7]. Third-line treatment refers to the treatment adopted after the failure of the second-line treatment. Generally, there are lesser drugs and effective treatment regimen for the third-line treatment, so the first-line treatment is the most crucial, which directly determines the prognosis of patient survival. Once the tumor resists to the first-line treatment, the subsequent treatment will obtain poorer effect, and therefore, it is necessary to actively explore highly efficient drugs used in the third-line treatment for prolonging the survival of NSCLC patients. In recent years, molecular targeted therapy has become a hot topic in treating NSCLC, which acts on a certain link of development and progression of tumor, such as inhibiting tumor angiogenesis and leading to tumor apoptosis. The advantage of molecular targeted therapy over conventional chemotherapeutic agents is that it does not cause toxic side effects such as myelosuppression and hair loss, so it is becoming the most acceptable treatment for medical workers and patients [8].

Anlotinib, a novel small-molecule and multitarget tyrosine kinase inhibitor independently developed in China, inhibits type III tyrosine kinase and platelet-derived growth factor receptor (PDGFR) to suppress tumor angiogenesis and growth, with the efficacy that has been proven in treating brain glioblastoma and metastatic renal cell carcinoma [9, 10]. Camrelizumab, a humanized monoclonal antibody extracted from the hamster ovary cell line by recombinant technique, can bind to programmed death receptor-1 (PD-1), block the binding of PD-1 and programmed death receptor ligand 1 (PD-L1), reactivate T cells, produce sustained antitumor effect, and inhibit tumor growth, which has been confirmed in primary liver cancer with lung metastasis [11]. At present, no report has been found on the application of anlotinib capsules combined with the PD-1 inhibitor (camrelizumab) in the third-line treatment of patients with advanced NSCLC. This study adopted the combined treatment to explore its application value by observing the clinical manifestations and clinical indexes of patients.

## 2. Materials and Methods

### 2.1. General Information

Eighty-eight patients with advanced NSCLC treated in the Oncology Department of our hospital from December 2018 to December 2019 were selected as research subjects and randomly and equally split into the single treatment group (STG) and combined treatment group (CTG). Patients or legal guardians signed informed consent and volunteered to participate in the study.

### 2.2. Inclusion and Exclusion Criteria

#### 2.2.1. Inclusion Criteria

The inclusion criteria were as follows: (1) all the enrolled patients met the diagnostic criteria of this disease in the *Diagnostic and Therapeutic Norms for Primary Lung Cancer (2018 edition)* [11], were confirmed by tissue biopsy and MRI with the clinical manifestations such as expectoration, dyspnea, and hemoptysis, and conformed to the stage IV staging criteria in *International Standards for Lung Cancer Staging (8th edition)* [12]; (2) the patients were no less than 18 years old, with the estimated survival period no less than 3 months; (3) the patients did not have contraindications in the drugs used in the study; and (4) the patients' physical condition allowed them to receive further treatment.

#### 2.2.2. Exclusion Criteria

The exclusion criteria were as follows: (1) patients with abnormal coagulation and a risk of major bleeding; (2) patients complicated with failure of organs such as the liver, kidney, and heart, requiring supportive treatment or rescue; (3) patients with uncontrolled hypertension; (4) patients with a history of other malignancies.

### 2.3. Methods

All patients were treated with anlotinib hydrochloride (manufacturer: Chia Tai Tianqing Pharmaceutical Group Co., Ltd.; NMPA approval no. H20180003; specification: 12 mg *∗* 7 capsules), with 12 mg/time and 1 time/d for 2 consecutive weeks, followed by 1 week of rest. A treatment cycle included 3 weeks. Patients were discontinued until the occurrence of disease progression, intolerant adverse events, death, or refusal of treatment [13]. The dosage was reduced to 10 mg/d if grade 3 and above of anlotinib-related adverse events occurred during treatment (including ① systolic blood pressure ≥180 mmHg; ② severe skin changes such as bleeding, edema, blister, ulcer, peeling, hyperkeratosis, obvious pain, and limited self-care ability; and ③ 24 h urine protein excretion ≥3.5 g) and to 8 mg/d if the patients remained intolerant. If still intolerant, the drug was discontinued.

CTG received anlotinib hydrochloride combined with camrelizumab. 200 mg of camrelizumab (manufacturer: Suzhou Sheng Diya Biomedical Co., Ltd.; NMPA approval no. S20190027; specification: 200 mg/vial) was injected by an intravenous drip, 200 mg/time, 1 time/3 weeks. A chemotherapy cycle included 3 weeks. Drug administration was discontinued until the progression of the disease or the patients were intolerant.

### 2.4. Observation Indexes

The objective efficacy evaluation of tumors was as follows. The lesion size of the patients was recorded according to the results of CT, MRI, and other imaging examinations, and the therapeutic effect was evaluated using Response Evaluation Criteria in Solid Tumors (RECIST) [14]. The efficacy was complete response (CR, disappearance of all target lesions completely after treatment), partial response (PR, reduction of lesions >50% and no new lesions), no change (NC, no significant improvement in clinical symptoms with tumor reduction between 25% and 50%), and progression of the disease (PD, tumor increase >25% or appearance of new lesions). Total effective rate = (CR + PR)/total number of cases × 100%; 5 ml of fasting elbow venous blood was collected after treatment and centrifuged at 3500 r/min for 10 min. The levels of serum carcinoembryonic antigen (CEA), neuron-specific enolase (NSE), and cytokeratin-19 fragment (CYFRA 21-1) were detected by electrochemiluminescence. All the detection instruments were Roche cobas e 411 automatic electrochemiluminescence immunoassay analyzer (manufacturer: Shanghai Mojin Medical Device Co., Ltd.) and matching reagents (manufacturer: Shanghai Univ Biotechnology Co., Ltd.).

The German version of the Cancer Fatigue Scale (CFS) [15] was for evaluating the fatigue degree after treatment, including 15 items such as body, activity, attention, memory, and emotion, with each item scoring 5 points, a total score of 75 points. Higher scores represented more severe fatigue.

Karnofsky Performance Status (KPS) [16] was used to evaluate the physical condition of both groups before and after treatment, with the specific scoring criteria in Table 1.

The incidence of adverse reactions in both groups during treatment was analyzed, including hypertension, hand and foot syndrome, anemia, reactive cutaneous capillary hyperplasia, chest pain, and hemoptysis.

### 2.5. Statistical Methods

The data were processed by SPSS 23.0 and graphed by GraphPad Prism 7 (GraphPad Software, San Diego, USA). Enumeration data were tested by *X*^2^ and expressed as *n* (%), while measurement data were tested by *t*-test and expressed as mean ± SD. When *P* < 0.05, the differences were statistically significant.

## 3. Results

### 3.1. Comparison of Baseline Data

No significant differences in baseline data such as sex ratio, average age, pathological types, and metastatic sites were observed between the two groups (*P* > 0.05; Table 2).

### 3.2. Comparison of Short-Term Efficacy

The total effective rate was remarkably higher in the CTG than in the STG (*P* < 0.05; Table 3).

### 3.3. Comparison of Serum Tumor Marker Levels

After treatment, the levels of various serum tumor markers in the CTG were obviously lower compared with the STG (*P* < 0.001; Figure 1).

### 3.4. Comparison of CFS Scores after Treatment

The average CFS score after treatment in the CTG was obviously lower compared with the STG (*P* < 0.001; Figure 2).

### 3.5. Comparison of KPS Scores after Treatment

The average KPS score after treatment was markedly higher in the CTG than in the STG (*P* < 0.001; Figure 3).

### 3.6. Safety Comparison

The total incidence of adverse reactions in the CTG was lower compared with the STG (*P* < 0.05; Table 4).

## 4. Discussion

The incidence of lung cancer is increasing in China, accounting for the first and second place in male and female tumors, making it one of the malignant tumors with the highest mortality. In the early stage, the tumor does not involve the trachea, pleura, and bronchial mucosa and surrounding blood vessels, so there will be no symptoms of cough, chest pain, and hemoptysis, and therefore, the diagnosis of lung cancer is delayed to a great extent. A survey [17] has revealed that 75% of NSCLC patients are in advanced stages at diagnosis and miss the best surgery time. Although the existing chemotherapy regimens can play a certain therapeutic effect, most patients cannot tolerate the serious adverse reactions, and advanced NSCLC patients with multiline chemotherapy failure are difficult to benefit from chemotherapy again. As a novel micromolecule multitarget TKI (tyrosine kinase inhibitor) independently developed in China, anlotinib capsules are convenient for oral administration, with little adverse reactions and good patient tolerance in clinical trials, which are expected to become the typical drug in the third-line treatment of NSCLC in China [18]. In a clinical study [19], 166 patients with advanced soft tissue sarcoma were treated with anlotinib, and the results showed that the 12-week disease progression-free rate was 68%, progression-free survival time was 5.6 months, and the overall median survival time was 12 months. Camrelizumab is a humanized monoclonal antibody obtained by the recombinant technique. Since this drug has shown good survival benefits in the single-arm phase II clinical trials of typical Hodgkin's lymphoma, it is used to treat recurrent or refractory classical Hodgkin's lymphoma after second-line systemic chemotherapy [20].

Among the treatment methods of various tumor diseases, the combined therapy has more advantages for patients. Lou et al. [21] pointed out in the study that the survival curves of patients treated with single drug and chemotherapy were crossed, suggesting that some patients cannot benefit from single-drug therapy. Visser et al. [22] found an obvious difference in the survival curves at the early stage between patients treated with combined therapy and those treated with monotherapy, demonstrating that the combined therapy is the better treatment pattern for cancer. In this paper, anlotinib capsules combined with the PD-1 inhibitor (camrelizumab) were adopted to treat advanced NSCLC, and the results demonstrated that the total clinical effective rate of the CTG was 93.18% (41/44), which was higher than 75.00% (33/44) of the STG, revealing that the combined treatment could significantly improve the efficacy of patients with advanced NSCLC compared with the simple treatment, with positive significance for prolonging the survival time and improving the prognosis. CYFRA 21-1 is an epithelial cell characteristic marker, mainly distributed in unilayer epithelial cells and pseudostratified epithelial cells, so this serum tumor marker is a good indicator of tumors of epithelial origin. Comparison of serum tumor marker levels after treatment in this study showed that the levels were lower in the CTG than in the STG (*P* < 0.001), suggesting that the combined treatment was more conducive to the treatment of patients with tumors. The presence of cancer fatigue is related to the course of the disease and chemotherapy on the one hand and the experience of persistent subjective fatigue on the other hand, which can not only lead to a decrease in the quality of life of patients but also promote the progression of the condition, leading to discontinue treatment. The study results confirmed that the mean CFS score after treatment was significantly lower in the CTG than in the STG (*P* < 0.001), indicating that the combination modality could reduce their cancer fatigue and contribute to the improvement of quality of life. In terms of adverse reactions, the PD-1 inhibitor (camrelizumab) not only benefits the majority of cancer patients but also brings immune-related adverse reactions because it can involve multiple systems in the human body [23]. Among them, reactive cutaneous capillary hyperplasia is the most common adverse drug reaction of camrelizumab, with the clinicopathologic features of dermal capillary increase and proliferation of capillary endothelial cells. Its current pathogenesis remains unclear, which may be due to the imbalance between angiogenesis promoters and inhibitors [24]. The study showed that only 3 patients had this symptom during treatment in the CTG but did not endanger life, and the patients recovered spontaneously after a period of drug withdrawal.

The study also has some limitations. For example, the limited number of cases and the small sample size may lead to bias in the experimental results. In addition, it is impossible to analyze the median survival period of patients and long-term efficacy of the combined treatment. Therefore, multicenter studies with a larger sample size are needed in the future to further provide the best treatment regime for NSCLC patients.

In conclusion, the combination of anlotinib capsules and PD-1 inhibitor (camrelizumab) is a reliable scheme in the third-line treatment of advanced NSCLC, which greatly reduces the serum tumor markers of patients, with high safety and clinical application value.

## Figures and Tables

**Figure 1:** Comparison of serum tumor marker levels after treatment (mean ± SD). (a) Comparison of CEA levels. The abscissa was STG and CTG, and the ordinate was the CEA level (ng/ml). The CEA levels in the STG and CTG were 76.26 ± 3.64 ng/ml and 44.35 ± 3.48 ng/ml.  ^*∗*^indicated a remarkable difference in the CEA levels between the two groups after treatment (*t* = 42.032, *P* < 0.001). (b) Comparison of CYFRA 21-1 levels. The abscissa was STG and CTG, and the ordinate was the CYFRA 21-1 level (ng/ml). The CYFRA 21-1 levels in the STG and CTG were 16.74 ± 1.35 ng/ml and 10.32 ± 1.28 ng/ml. ^*∗∗*^indicated a remarkable difference in the CYFRA 21-1 levels between the two groups after treatment (*t* = 22.891, *P* < 0.001). (c) Comparison of NSE levels. The abscissa was STG and CTG, and the ordinate was the NSE level (ng/ml). The NSE levels in the STG and CTG were 24.16 ± 2.43 ng/ml and 12.54 ± 2.56 ng/ml. ^*∗∗∗*^indicated a remarkable difference in the NSE levels between the two groups after treatment (*t* = 21.837, *P* < 0.001).

**Figure 2:** Comparison of CFS scores after treatment (mean ± SD). Note: the abscissa was STG and CTG, and the ordinate was the CFS score (points). The average CFS scores after treatment in the STG and CTG were 69.75 ± 3.38 and 55.16 ± 7.09. ^*∗*^indicated an obvious difference in the average CFS scores after treatment between the two groups (*t* = 12.322, *P* < 0.001).

**Figure 3:** Comparison of KPS scores after treatment (mean ± SD). Note: the abscissa was STG and CTG, and the ordinate was the KPS score (points). The average KPS scores in the STG and CTG were 66.96 ± 3.21 and 79.02 ± 1.86.  ^*∗*^ indicated a remarkable difference in the average KPS scores between the two groups after treatment (*t* = 21.563, *P* < 0.001).

**Table 1:** Karnofsky behavior scoring criteria.

Physical condition	Points
Normal condition, no symptoms or signs	100
The patients could carry out normal activities, with mild symptoms and signs	90
The patients could carry out normal activities reluctantly, with some symptoms and signs	80
The patients could take care of themselves in daily life, but could not maintain normal life or activities	70
Sometimes, the patients needed help, but could generally take care of themselves	60
The patients needed others to look after them	50
The patients could not take care of themselves and needed special care	40
The patients could not take care of themselves at all	30
The patients had aggravated condition and required inpatient treatment	20
The patients were critically ill and close to death	10
Death	0

**Table 2:** Comparison of baseline data (*n* = 44).

Items	STG	CTG	*X* ^2^/*t*	*P*
Gender			0.188	0.665
Male	27 (61.36%)	25 (56.82%)		
Female	17 (38.64%)	19 (43.18%)		
Average age (mean ± SD, years old)	64.38 ± 7.28	64.56 ± 7.24	0.116	0.908
BMI (mean ± SD, kg/m^2^)	21.25 ± 1.26	21.32 ± 1.23	0.264	0.793
Pathological types				
Adenocarcinoma	24 (54.55%)	26 (59.09%)	0.185	0.667
Squamous cell carcinoma	17 (38.64%)	14 (31.82%)	0.448	0.503
Others	3 (6.82%)	4 (9.09%)	0.155	0.694
Metastatic sites				
Liver	12 (27.27%)	10 (22.73%)	0.246	0.620
Pleura	8 (18.18%)	11 (25.00%)	0.612	0.434
Lymph nodes	19 (43.18%)	16 (36.36%)	0.441	0.507
Bones	5 (11.36%)	7 (15.91%)	0.389	0.533
Smoking history			0.279	0.597
Yes	34 (77.27%)	36 (81.82%)		
No	10 (22.73%)	8 (18.18%)		
Drinking history			0.196	0.658
Yes	29 (65.91%)	27 (61.36%)		
No	15 (34.09%)	17 (38.64%)		
Marital status				
Married	40 (90.91%)	39 (88.64%)	0.124	0.725
Unmarried	1 (2.27%)	3 (6.82%)	1.048	0.306
Divorced	3 (6.82%)	2 (4.55%)	0.212	0.645
Education level				
University	6 (13.64%)	4 (9.09%)	0.451	0.502
Middle school	12 (27.27%)	16 (36.36%)	0.838	0.360
Primary school	26 (59.09%)	24 (54.55%)	0.185	0.667
Residence			0.049	0.826
Urban area	17 (38.64%)	16 (36.36%)		
Rural area	27 (61.36%)	28 (63.64%)		

**Table 3:** Comparison of short-term efficacy (*n* (%)).

Group	*n*	CR	PR	NC	PD	Total effective rate
CTG	44	25 (56.82%)	16 (36.36%)	2 (4.55%)	1 (2.27%)	93.18% (41/44)
STG	44	19 (43.18%)	14 (31.82%)	7 (15.91%)	4 (9.09%)	75.00% (33/44)
*X* ^2^						5.436
*P*						<0.05

**Table 4:** Comparison of the incidence of adverse reactions (*n* (%)).

Group	Hypertension	Hand-foot syndrome	Anemia	Reactive cutaneous capillary hyperplasia	Chest pain	Hemoptysis	Total incidence
STG	3 (6.82)	3 (6.82)	2 (4.55)	0 (0.00)	2 (4.55)	3 (2.27)	29.55% (13/44)
CTG	1 (2.27)	0 (0.00)	1 (2.27)	3 (6.82)	0 (0.00)	0 (0.00)	11.36% (5/44)
*X* ^2^							4.470
*P*							<0.05

## Data Availability

The data used to support the findings of this study are available from the corresponding author upon reasonable request.
